# Analysis of the Effect of DPL Combined with Clarithromycin in the Therapy and Improvement of Rosacea

This article has been retracted.

**DOI:** 10.1155/2022/9437697

**Published:** 2022-08-19

**Authors:** Fang Yan, Chao Peng

**Affiliations:** Department of Dermatology, People's Hospital of Dongxihu District, Hubei 430040, China

## Abstract

Rosacea is a chronic inflammatory skin disease with a high incidence, and it leads to negative emotions such as inferiority complex, increased psychological pressure, and a greatly reduced quality of life. In order to investigate the clinical efficacy of DPL combined with clarithromycin in the treatment and improvement of rosacea. 86 patients with rosacea were selected and randomly divided into the control group and study group according to the random number table method. The results show that the combination of DPL and clarithromycin in the treatment of rosacea patients can effectively improve the clinical symptoms of patients, improve the therapeutic effect, and the incidence of adverse reactions is low, which ensures that the patients have a good prognosis, which is worthy of clinical application.

## 1. Introduction

Rosacea is a chronic inflammatory skin disease with a high incidence. The age of the patients is usually between 20 and 50 years old, but children and the elderly can also develop the disease because the disease is mainly manifested as paroxysmal flushing or persistent flushing. It is accompanied by erythema, papules, pustules, and telangiectasia, etc., and it occurs on the facial skin, which may affect the patient's face, which may lead to negative emotions such as inferiority complex, increased psychological pressure, and greatly reduced quality of life. It is not conducive to patients' daily lives and social activities. The etiology and pathogenesis of rosacea are complex and are related to Propionibacterium acnes infection, abnormal androgen secretion, strong sebum secretion, and other factors. In addition, genetic factors, neuroimmune dysfunction, etc., may also lead to rosacea [1, 2]. The commonly used clinical treatment of rosacea is oral medicine or external medicine, which has antibacterial and anti-inflammatory effects. However, the effect of simple drugs is not good, the patient's tolerance to drugs is gradually improved, and the patient's compliance is not high, so it is difficult to achieve a good treatment effect. In recent years, narrow-spectrum intense pulsed light (Dye pulsed light, or DPL) has become the main physical modality used in the clinical treatment of rosacea and is more easily accepted by patients. DPL can accurately deliver intense pulsed light therapy spectrum to the lesion area, which is precise and targeted and can effectively improve vasodilation, papules, pustules, and erythema caused by rosacea. The research team led by Zhang Tianlong confirmed that the combined use of DPL can effectively improve rosacea based on the use of low-dose minocycline hydrochloride [3]. However, there are few domestic and foreign scholars' studies on the therapeutic effect of DPL combined with clarithromycin on rosacea. Therefore, this study selected 86 patients with rosacea to study and analyze the clinical efficacy of DPL combined with clarithromycin in the treatment of rosacea.

The rest of this paper is organized as follows: Section 2 discusses related research and analysis, followed by the patients' information and research methods in Section 3. The comparative analysis and data statistics are discussed in Section 4.  Section 5 concludes the paper with a summary and future research directions.

## 2. Related Research and Analysis

As a chronic inflammatory skin disease, rosacea mainly occurs on the face, which affects the sufferer's appearance and affects the sufferer's studies, work, and life [4]. Therefore, early diagnosis and therapy should be carried out. However, the etiology and pathogenesis of the disease involve a variety of factors, and there is no unified conclusion yet. The commonly used method for the therapy of rosacea is to administer anti-inflammatory drugs and carry out anti-inflammatory and antibacterial therapy. In domestic clinical therapy, tetracycline antibiotics or macrolide antibiotics are more commonly used [5]. However, some studies show that although the use of simple drugs in the clinical therapy of rosacea has a certain effect, the effect is poor, so it is necessary to combine physical therapy such as DPL [6]. This study shows that DPL combined with clarithromycin has a good effect on the therapy and improvement of rosacea.

Narrow-spectrum intense pulsed light (DPL) therapy, as a phototherapy method, should be used in combination with other drugs without photosensitivity, so this study selected clarithromycin combined with DPL therapy [7]. Clarithromycin is a kind of macrolide antibiotic. It has no photosensitivity, and clarithromycin can effectively target anaerobic infection. It can also inhibit Gram-positive bacteria and can play an antibacterial and role[8, 9].

Scholars such as Qiu Wenyuan find that clarithromycin can significantly improve the inflammatory response of rosacea and relieve the papules and erythema caused by rosacea, which is similar to the results in [10]. The results of this study showed that after treatment, the symptom scores of both groups decreased, and the study group is significantly lower than the control group (*P* < 0.05); the clinical efficacy of the study group was better than that of the control group, and the treatment effective rate of the study group reached 74.42%, which is significantly higher compared to the control group, and the difference is statistically significant (*P* < 0.05). Analysis of its mechanism may suggest that clarithromycin has an anti-inflammatory effect. When clarithromycin enters the body, it can penetrate the cell wall of bacteria, inhibit the synthesis of bacterial ribosomal 50*S* subunit protein, and finally inhibit the production of bacteria to achieve the purpose of anti-inflammatory [11]. After the inflammation is reduced or eliminated, the erythema fades, the papules subside, and the skin condition significantly improves.

Clarithromycin alone can be effective for papules and pustules caused by rosacea, but it is less effective for erythema and telangiectasia. Therefore, it is necessary to strengthen the therapy effect by other means, such as therapy in combination with DPL. DPL therapy has the advantages of low pain, good safety, short recovery time, and high sufferer compliance, and has become the preferred physical solution for the therapy of rosacea. The results of this study show that after the combined therapy of DPL and clarithromycin in sufferers with rosacea, the GAGS score of the sufferers has notoriously decreased, and the acne is notoriously improved, and the disparity is statistically extensive (*P* < 0.05). The score of the study set is notoriously cut down than that of the contrast set, *P* < 0.05, and the disparity is statistically extensive. There is no extensive disparity in the incidence of adverse reactions between the two sets (*P* > 0.05). Analysis of its mechanism may be that DPL combined with clarithromycin therapy greatly enhances the therapeutic effect of rosacea. As a narrow-spectrum intense pulsed light, DPL can target the diseased tissue, but has no effect on the adjacent normal tissue, which makes the therapy more targeted and can effectively treat and improve rosacea [12, 13]. Contrast with intense pulsed light (IPL), DPL is more accurate, with smaller wounds and less consumables after therapy. DPL also has fewer adverse reactions during therapy and is safe. The postoperative wound healing time is short, the therapy efficacy is greatly improved, and the impact on the sufferer's social life and work is small, so that the sufferer's quality of life is greatly improved [14, 15].

Due to the high selectivity of photothermolysis, DPL therapy makes the photon energy highly concentrated, and hemoglobin absorbs the light energy and converts it into heat energy. The purpose of eliminating or reducing inflammation. The combination of clarithromycin also inhibits the production of inflammatory factors and reduces the immune system response to limit the production of inflammation. In addition, DPL combined with clarithromycin can effectively relieve or eliminate erythema, papules, etc. on the sufferer's face, repair damaged skin, and help rebuild the skin barrier. The therapy method is quick and effective, the sufferer's compliance and enthusiasm are further enhanced, the sufferer's self-confidence is also notoriously improved, the negative emotions are eliminated, and the quality of life is greatly improved.

## 3. Patients Information and Research Methods

### 3.1. General Information

A total of 86 patients with rosacea treated in our hospital from December 2019 to August 2021 are selected as the research subjects, and the patients are randomly divided into the control group of 43 cases and the study group of 43 cases, aged 23 to 67 years old, by random number table method. The mean age is (55.21 ± 6.53) years old. There is no extensive disparity in general data such as gender composition and course of disease between the two sets (*P* > 0.05). All sufferers participating in this study signed informed consent.

Inclusion criteria: Firstly, meet the diagnostic criteria for rosacea. Secondly, age > 18 years, no gender restriction. Thirdly, normal liver function. Fourthly, it is not dyslexia. Finally, it is no treatment for 2 weeks before treatment of any other treatment.

Diagnostic criteria for rosacea: erythematous papules on the nose or on both sides of the nose. Generally, there are three clinical stages: the erythematous stage is mainly flushing with telangiectasia. The popular stage is the appearance of scattered rice grain-sized papules or small pustules mixed with small pustules on the basis of the flushing, but no comedies. In hypertrophy and hyperplasia, the surface is uneven like a rhinophyma. Generally, no symptoms of discomfort. Histopathological examination mainly shows telangiectasia, sebaceous gland hyperplasia, or hyperplasia of connective tissue and sebaceous glands.

### 3.2. Methods

The control group is given oral Clarithromycin Tablets, specification: 250 mg/tablet, twice a day, 1 tablet each time, for 6 weeks. At the same time, patients should be instructed to avoid greasy and spicy food, avoid sunlight and sunscreen, reasonably guide negative emotions, and maintain a good mood.

Inclusion criteria: Firstly, meet the diagnostic criteria for rosacea. Secondly, age > 18 years, no gender restriction. Thirdly, normal liver function. Fourthly, it is not dyslexia. Finally, it is no treatment for 2 weeks before treatment of any treatment.

The patients in the study group received DPL treatment on the basis of the control group [15]. The DPL used is Feidun's black gold laser photonic workstation DPL500 hand tool, wavelength 500 ∼ 600 nm, VL mode, pulse width 10 ∼ 15 ms, energy density: 8 ∼ 15 J/cm^2^. The specific treatment methods are as follows: Firstly, before treatment, the patient is informed of the precautions and related risks of the treatment, and the patient should sign the informed consent. Secondly, before treatment, the patient should clean the face, apply medical cold gel evenly, and cover it with a visor. Thirdly, adjust the corresponding treatment parameters according to the actual conditions of the patient's skin lesion color, skin tone, tolerance, etc. For the first treatment, a spot test should be performed and the parameters should be adjusted. Adjust the treatment parameters in time according to the patient's condition to ensure the effectiveness of the treatment. Fourthly, when the patient's skin erythema is slightly deepened and the blood vessels are blurred or disappear, the treatment can be stopped. Finally, the medical cold gel should be cleaned after surgery, and the treatment for cold compresses should be applied to the area, and epidermal growth factor can be applied after surgery to promote wound healing.

After DPL therapy, sufferers should avoid light, take sun protection measures, keep a light diet, and avoid scratching the affected area. The therapy is done once every 4 weeks, with 3 therapies as a therapy cycle.

### 3.3. Observation Indicators and Evaluation Criteria

The differences in scores of erythema, telangiectasia, papules, pustules, and pruritus before and after treatment are compared to evaluate the therapeutic effect. Each item is scored on a scale of 0 to 3, and the lower the score, the milder the patient's symptoms. In order to compare the difference in clinical efficacy between the two groups, the criteria were as follows: the recovery reduction of facial erythema and telangiectasia was 90%. Facial erythema and telangiectasia were significantly effective, reducing by 60% to 89%. Facial erythema and telangiectasia were reduced by 25% to 59%. The ineffective rate and improvement rate of facial erythema and telangiectasia were less than 25%. Effective rate = (number of cured cases + number of markedly effective cases)/total number of cases × 100%. The differences in the global acne grading system (GAGS) scores before and after treatment are compared [8]. The facial skin lesions of the two groups of patients are recorded before and after treatment, and the facial skin lesions are papules and pustules. Using the GAGS scoring system, it is divided into 6 areas: the forehead (2 points), the right cheek (2 points), the left cheek (2 points), the nose (1 point), the chin (1 point), the chest, and the upper back (3 points). Skin lesion score: 1 point for ≥1 acne, 2 points for ≥1 papule, 3 points for ≥1 pustule, and 4 points for ≥1 nodule. The regional score = site score × skin lesion score, each area. The sum of the scores is the GAGS composite score. The disparities in the scores of quality of life between the two sets are contrast, and the dermatology life quality index (DLQI) is used to test. Using a 4-level scoring method, according to the standard score of “none,” “less,” “severe,” and “very serious,“ respectively, 0, 1, 2, and 3 points, with a full score of 15 points. The lower the score, the better the patient's quality of life. Compared to the differences in the occurrence of adverse reactions, including redness, hyperpigmentation, and gastrointestinal reactions the recurrence rate after 6-month follow-up between the two sets is at contrast.

### 3.4. Statistical Processing

In this study, all the data are organized, and a corresponding database is established for it, and all the databases are entered into SPSS 26.0 for data processing, and the measurement data is tested for normality. The independent sample *t*-test is used for the data between multiple sets, the paired sample *t*-test is used for the data within the set, and the Mann–Whitney *U* test is used for non-normality. The rate of enumeration data is expressed as %, and the test is *χ2* (*P* < 0.05), the data are considered to be data. The disparity is statistically extensive.

## 4. The Case Analysis and Comparison

### 4.1. Comparison of Differences in Symptom Scores before and after Treatment

Before treatment, there was no significant difference in the symptom scores of erythema, telangiectasia, papules, pustules, and pruritus between the two groups (*P* > 0.05). After treatment, the symptom scores of the two groups are decreased, and the study group is significantly lower than the control group (*P* < 0.05). The difference is statistically significant, as shown in Table 1.

### 4.2. To Compare the Disparities in Clinical Efficacy between the Two Sets of Sufferers

Contrast with the contrast set, the therapy effect of the study set is notoriously better than that of the contrast set, and the therapy effective rate reached 74.42%, and the disparity is statistically extensive (*P* < 0.05), as shown in Table 2.

### 4.3. Contrast of the GAGS Scores before and after Therapy

Table 3 shows the GAGS scores of the two sets are notoriously decreased in contrast with those before therapy (*P* < 0.05).

The disparity is statistically extensive, as shown in Figure 1.

### 4.4. Contrast of Disparities in Quality of Life Scores between the Two Sets of Sufferers

In comparison with before therapy, the DLQI scores of the two sets of sufferers after therapy notoriously decreased, *P* < 0.05. The disparity is statistically extensive, as shown in Table 4.

### 4.5. Contrast of the Disparities in the Occurrence of Adverse Reactions

Adverse reactions occurred in 3 patients in the research group. The research group included 1 patient with redness and swelling, which is relieved by cold compress and subsided after one week, 1 patient had local hyperpigmentation, which subsided at the follow-up 6-month later, and 1 patient had gastrointestinal reaction without pigment, as shown in Table 5.

There are 2 cases of adverse reactions in the control group, all of which are gastrointestinal reactions without redness, hyperpigmentation, and hypopigmentation. The gastrointestinal reactions in the two groups are tolerated, and there is no significant difference in the incidence of adverse reactions (*P* > 0.05), as shown in Figure 2.

### 4.6. Contrast of the 6-Month Recurrence Rate of the Two Sets of Sufferers

Both sets of sufferers are followed up for 6 months, and the follow-up deadline is February 2022. There are 12 sufferers in the contrast set who are readmitted to the hospital for therapy, and the recurrence rate is 27.91% (12/43), which is notoriously higher compared to the 2 sufferers in the study set who had recurrence. The recurrence rate is 6.98% (3/46), and the disparity is statistically extensive (*χ*2 = 8.425, *P* < 0.05), as shown in Figure 3.

## 5. Conclusions

In conclusion, DPL combined with clarithromycin has an obvious curative effect on the treatment and improvement of rosacea, with high safety and few adverse reactions and can effectively improve the clinical symptoms and prognosis quality of life of patients. Expand the sample size to further verify the effectiveness of this method in clinical treatment.

## Figures and Tables

**Figure 1:** Contrast of the GAGS scores before and after therapy in two sets of sufferers.

**Figure 2:** Comparison of adverse reactions in the two groups of patients.

**Figure 3:** Contrast of the 6-month recurrence rate in the two sets of sufferers.

**Table 1:** Comparison of symptom scores in the two groups before and after treatment (points, $\bar{x}\pm s$).

Set	Number of case (*n*)	Erythema		Telangiectasia		Papules		Pustules		Itching	
		Before therapy	After treatment	Before therapy	After treatment	Before therapy	After treatment	Before therapy	After treatment	Before therapy	After treatment
Research set	43	2.52 ± 0.97	1.38 ± 0.56	2.53 ± 1.03	1.23 ± 0.87	2.71 ± 1.23	1.52 ± 0.93	2.62 ± 0.99	1.27 ± 0.86	2.77 ± 1.06	1.19 ± 0.85
Contrast set	43	2.57 ± 0.65	0.83 ± 0.33	2.61 ± 1.10	0.75 ± 0.43	2.74 ± 1.19	1.03 ± 0.72	2.59 ± 1.12	0.88 ± 0.37	2.67 ± 0.98	0.67 ± 0.29
*t*		1.237	6.031	0.596	7.836	0.715	7.182	0.935	6.953	0.893	9.523
*P*		0.138	<0.001	0.512	<0.001	0.493	<0.001	0.325	<0.001	0.421	<0.001

**Table 2:** Contrast of clinical efficacy between the two sets of sufferers (*n*/%).

Set	Number of cases	Get well	Effective	Progress	Invalid	Efficient (%)
Research set	43	19 (44.19)	13 (30.23)	9 (20.93)	2 (4.65)	74.42
Contrast set	43	6 (13.95)	8 (18.60)	19 (44.19)	10 (23.26)	32.56
*χ* ^2^						11.39
*P*						0.027

**Table 3:** Contrast of the GAGS scores between the two sets before and after therapy (points, $\bar{x}\pm s$).

Set	Number of cases (*n*)	Before therapy	After therapy	*t*	*P*
Research set	43	37.64 ± 6.82	11.03 ± 7.23	16.852	0.019
Contrast set	43	36.29 ± 7.31	20.58 ± 5.47	8.623	0.037
*t*		1.349	5.462		
*P*		0.062	<0.001		

**Table 4:** Contrast of the DLQI scores between the two sets before and after therapy (points, $\bar{x}\pm s$).

Set	Number of cases (*n*)	Before therapy	After therapy	*t*	*P*
Research set	43	12.68 ± 2.35	2.08 ± 1.03	15.236	0.021
Contrast set	43	12.53 ± 2.47	5.62 ± 2.21	7.935	0.038
*t*		1.263	3.519		
*P*		0.177	<0.001		

**Table 5:** Comparison of the adverse reactions in the two groups of patients (*n*/%).

Set	Number of cases	Redness	Pigmentation	Hypopigmentation	Gastrointestinal reactions	Total incidence
Research set	43	1	1	0	1	3
Contrast set	43	0	0	0	2	2
*χ* ^2^						0.965
*P*						0.413

## Data Availability

The simulation experiment data used to support the findings of this study are available from the corresponding author upon request.
